# Circ_0001897 regulates high glucose-induced angiogenesis and inflammation in retinal microvascular endothelial cells through miR-29c-3p/transforming growth factor beta 2 axis

**DOI:** 10.1080/21655979.2022.2070997

**Published:** 2022-05-05

**Authors:** Yudan Gong, Xinze Li, Liuyi Xie

**Affiliations:** a Department of Ophthalmology, Beilun People’s Hospital, Ningbo, China; b Department of Traditional Chinese Medicine, Beilun People’s Hospital, Ningbo, China

**Keywords:** Circ_0001897, mir-29c-3p, diabetic retinopathy, TGFB2

## Abstract

Diabetic retinopathy (DR) has become the leading cause of blindness among adults at working age. Previous studies have implicated circ_0001897 in the development of DR. In this study, we investigated the functional roles and mechanisms of circ_0001897 in high glucose-induced angiogenesis and inflammation. Peripheral blood samples from DR patients and healthy controls were collected to examine circ_0001897 expression, which demonstrated a significant upregulation of circ_0001897 in DR patients. To investigate the functional role and mechanisms of circ_0001897, human retinal microvascular endothelial cells (HRECs) were treated with high glucose (HG) to establish an *in vitro* DR model of endothelial cells. HG treatment induced the upregulation of circ_0001897 in HRECs, and enhanced cell proliferation, inflammatory responses, as well as *in vitro* angiogenesis. Circ_0001897 knockdown significantly attenuated the cell proliferation, inflammatory responses, and angiogenesis induced by HG treatment. Mechanistically, circ_0001897 sponged and inhibited the activity of mir-29c-3p, which in turn regulates the downstream target transforming growth factor beta 2 (TGFB2). The effects of circ_0001897 knockdown could be rescued by mir-29c-3p inhibitor or TGFB2 overexpression. Collectively, our data demonstrated the novel role of circ_0001897/mir-29c-3p/TGFB2 axis in regulating HG-induced inflammation and angiogenesis of HRECs. These findings suggest that targeting circ_0001897 could serve as an intervention strategy to ameliorate DR.

## Highlights

- Circ_0001897 is upregulated in DR patients and high glucose (HG)-induced HRECs;
- Silencing circ_0001897 attenuated HG-induced inflammation and angiogenesis in HRECs;
- Circ_0001897 sponges mir-29c-3p and regulates TGFB2 expression in HRECs.

## Introduction

Diabetes mellitus (DM) is a worldwide chronic disease characterized by hyperglycemia and neurovascular damages caused by insulin deficiency or insulin insensitivity [1]. Among the complications associated with DM, diabetic retinopathy (DR) is one of the most common and serious complications in diabetic patients, which can eventually lead to blindness [2,3]. The incidence of DR is escalating with the increasing diagnosis of diabetic patients worldwide [4,5]. DR has also been recognized as a major risk factor for blindness in the working population [6]. Blood vessel dysfunction due to retinal revascularization and inflammation in DR is considered as the main defect resulting in undesired fluid accumulation in the retina and visual impairment [7]. Currently, there is no effective treatment for DR and the underlying mechanisms of retinal dysfunction in DR patients are not fully understood.

In eukaryotes, circular RNAs (circRNAs) are produced by reverse splicing of exons in mRNA precursors of coding genes. They are a novel class of non-coding RNAs characterized by covalent bonding of 3’ and 5’-terminal, and widely implicated in the regulation of cell differentiation, apoptosis, proliferation, and autophagy [8]. Accumulating evidence shows that circRNAs play important roles in the development of human diseases, such as cancer and cardiovascular diseases [9,10]. Moreover, compared to other non-coding RNAs, such as miRNAs and long non-coding RNAs (lncRNAs), circRNAs have greater potential as diagnostic or prognostic biomarkers [10]. The dysregulation of circRNAs has been also reported in DM and DR. For example, circHIPK3 regulates gene programs in β-cell by inhibiting mir-121-3p and mir-338-3p [11]. Peripheral blood circRNAs can be used as diagnostic markers for prediabetes and type 2 diabetes mellitus (T2DM), with a sensitivity of 75% and a specificity of 79% [12]. A recent gene expression profiling analysis of circRNAs in between diabetic retinopathy and non-diabetes mellitus patients showed that circ_0001897 was upregulated in the retina of DR patients [13]. However, the functional engagement and mechanisms of circ_0001897 in DR progression are unclear.

MicroRNAs (miRNAs) are short, single-stranded RNAs that mainly bind to the 3’ untranslated region (3’ UTR) of target mRNAs and inhibit gene expression by inducing mRNA degradation or interfering the translation [14,15]. MiRNAs can regulate a wide spectrum of cellular and biological processes, including proliferation, apoptosis, differentiation, secretion of inflammatory cytokines, tumorigenesis, organogenesis, hematopoiesis, and antiviral innate immune responses [16]. Recent studies have implicated a large number of miRNAs in the regulation of diabetes and its complications. For instance, the abnormal expression of mir-200a [17], mir-200b [18] and mir-200c [19] in the retina of diabetic patients/rats suggests that the mir-200 family contributes to the pathogenesis of DR. In addition, a recent study revealed that mir-29c-3p is downregulated in patients with DR, which may serve as a risk factor for DR [20].

It was reported that the abnormal secretion of transforming growth factor β2 (TGFB2) contributes to the pathogenic defects in the retina of DR [21,22]. However, the mechanisms regulating TGFB2 expression in DR is not yet understood. Since circ_0001897 was upregulated in the retina of DR patients [13], but its roles and mechanisms in DR remain to be studied, in this study we aim to investigate the functional roles and mechanisms of circ_0001897 in DR and identify the downstream targets. We established an *in vitro* DR model of endothelial cells by treating human retinal microvascular endothelial cells (HRECs) with high glucose (HG). Using this cell model, we evaluated the functional engagement of circ_0001897 in HG-induced inflammatory responses and angiogenesis, and identified miR-29c-3p/TGFB2 axis as the downstream mediators of circ_0001897.

## Materials and methods

### Clinical samples

The peripheral blood samples of 22 DR patients and 20 normal subjects were collected at the department of Ophthalmology, Beilun People’s Hospital, Ningbo, China. The blood samples were snap-frozen in liquid nitrogen and stored at −80 degree freezer until further analysis. This study was approved by the Ethics Committee of Beilun People’s Hospital at Ningbo. The clinical parameters of the subjects were summarized in Supplementary Table S1.

### Cell culture

Human retinal microvascular endothelial cells (HRECs) were purchased from the Shanghai Institutes for Biological Sciences of the Chinese Academy of Sciences. These cells were cultured in endothelial cell medium with 1% endothelial cell growth supplement (ScienCell) and 5% FBS (ScienCell, USA) in a humidified incubator with 5% CO_2_ at 37°C. For high glucose induction, HRECs cells were treated with different concentrations of glucose (15, 25, 35 mmol/L), while the control group was supplied with normal glucose (5.5 mmol/L).

### Cell transfection

MiR-29c-3p mimic was used to overexpress miR-29c-3p in HRECs, and miR-NC served as negative controls. MiR-29c-3p inhibitor (anti-miR-29c-3p) was used to suppress miR-29c-3p, with NC inhibitor as control. Circ_0001897 siRNA was used to knockdown circ_0001897 expression in HRECs, with si-NC as the control. The full length of TGFB2 cDNA was constructed into pcDNA3.1 vector for overexpression, and blank pcDNA3.1 was used as control.

Cell transfection was performed using Lipofectamine® 3000 reagent (Thermo Fisher Scientific, L3000001). In 6-well plates, 60% confluent cells were transfected with 100 nM of microRNA mimic/inhibitor or 6 μg of pcDNA3.1-TGFB2 plasmid according to manufacturer’s instruction. Briefly, cells were seeded in 6-well plates at a density of 5x10^5 cells/well. Twenty-four hours later, each molecule was added into 100 µl Opti-MEM® I Reduced-Serum Medium (Invitrogen, Carlsbad, CA, USA, #31985062), and then 6 µL Lipofectamine 3000 reagent was added for 10 min incubation at room temperature. The mixture was added to the cell drop wise and the transfected cells were subjected to subsequent analysis 48 hours post-transfection [11].

### RT-qPCR

Total RNA was extracted from collected peripheral blood samples or from cultured HRECs using Trizol reagent according to the manufacturer’s instructions. The reverse transcription was performed with TransScript Green miRNA RT SuperMix (Transgen Biotech, Beijing, China), and the product was quantified using SYBR-Green PCR Master Mix Kit (Applied Biosystems, USA) on a 7900HT Fast Real-Time System (Applied Biosystems). The relative expression level of circ_0001897, miR-29c-3p and TGFB2 were calculated using 2 ^−ΔΔCt^ method and GAPDH served as the endogenous control [17]. All primer sequences were synthesized and purchased from Shanghai Sangon Biotechnology Co., Ltd. (Shanghai, China):

Circ_0001897, F-5'-CTGCCTACTCTTGCTCGTGG-3', R-5'-CAAAGCATA TGTGCG AGAGT-3'; miR-29c-3p, F-5'-GCTATCATATGTAGTTCGATATG-3'; R 5'-CTACACTCGCAGAGCTGTC-3'; TGFB2, F 5'-CCATCCCGCCCACTTTCTAC −3', R 5'-AGCTCAATCCGTTGTTCAGGC −3'.

### RNase R treatment

RNase R (TaKaRa, Maebashi, Japan) was used to degrade linear RNA. The RNA extraction sample was divided equally into two portions: one was used for RNase R digestion (RNase R group: treated with 10 unit of RNase R), and the other was used as control (Mock group: treated with equal volume of RNase-free water). The two portions of samples were incubated at 37°C for 25 min. The relative amount of GAPDH mRNA and circ_0001897 in each sample was detected by RT-qPCR [13].

### CCK‑8 proliferation assay

Cell proliferation of HRECs was examined using Cell Counting Kit-8 (Dojindo, Kumamoto, Japan). HRECs after the transfection were inoculated into 96-well plates at a density of 5000 cells per well. Cells were treated with HG (25 mmol/L) for 48 h and 10 μL of CCK-8 solution was added to the cell culture for 4 h incubation. The light absorption value (OD value) in each condition was captured at 450 nm wavelength on a Synergy H1 microplate reader (Winooski, Vermont, USA) [18].

### Luciferase reporter assay

To demonstrate the functional interaction, the sequence containing the wild-type binding sites or the sequence with mutated-binding sites were cloned into the PmirGLO firefly luciferase reporter (Promega, E1330). The reporter and Renilla luciferase (hRlucneo) control plasmid were co-transfected into cells in the presence of miR-29c-3p mimic or miR-NC in a 24-well plate (1 × 10^5 cells/well) using Lipofectamine 3000 reagent. 48 h after the transfection, the PierceTM Renilla-Firefly Luciferase Dual Assay Kit was used to determine the luciferase activities (Thermo Fischer Scientific, USA). The firefly luciferase activity in each sample was normalized to the activity of the control Renilla luciferase [17].

### RNA pull-down experiment

HREC cells lysates were collected by IP lysis buffer (Beyotime, P0013. Shanghai, China) and were incubated biotinylated miR-29c-3p oligo and miR-NC control oligos. 10% of the lysates was saved as the input. The mixture was further incubated with 100 μL M-280 streptavidin magnetic beads (Sigma-Aldrich, 11205D) at 4°C for 4 h. A magnetic bar was used to pull down the magnetic beads, and the beads were washed 4 times with lysis buffer. Both the input and samples in the beads from the pull-down were purified with Trizol reagent and analyzed by RT-qPCR [18].

### Western blot

Total protein was extracted from cell culture using RIPA lysis buffer containing protease inhibitor cocktail (Thermo Fisher Scientific 78429, Waltham, MA, USA). Cells suspended in RIPA buffer were lysed on ice for 10 min and the lysates were centrifuged at 14,000 rpm for 10 min. The supernatant containing total protein was quantified by a BCA Protein assay kit (Beyotime Biotechnology P0009; Shanghai, China). 10 µg of protein sample was mixed with SDS loading buffer and separated in 10% sodium dodecyl sulfat–polyacrylamide gel electrophoresis (SDS–PAGE) gel. The separated protein bands were transferred to polyvinylidene fluoride (PVDF) membranes, and the membranes were blocked with 5% skim milk in Tris-buffered saline Tween-20 (TBST) buffer for 1 h. The membrane was incubated with primary antibodies overnight at 4°C: anti-TGFB2 (1:2000, Abcam Ab9758) and anti-GAPDH (1:1000, Abcam Ab70699). After washing with TBST buffer, the membrane was incubated with HRP-conjugated secondary antibody (1:3000; Cell signaling #7074, MA, USA) at room temperature for 1 hour. After washing, the protein bands were developed using the EZ-ECL Chemiluminescence Detection kit (Pierce, Rockford, IL) and photographed on a gel imager system (Bio-Rad, Hercules, CA, United States). The densitometry analysis was performed with Image J software (Bethesda, MD, USA),with GAPDH as the loading control [18].

### Cell migration assay analysis

The transwell migration assay was carried out using transwell upper chamber (Corning, NY, USA, #3401) without Matrigel. 100 μl of cell suspension containing 1 × 10^4^ cells in serum-free medium was added to the upper chamber of the transwell, and 600 μL of 10% serum-containing medium was added to the lower chamber. After 48 h, the culture medium was discarded and the cells were fixed with 4% paraformaldehyde at room temperature for 10 min and stained with 0.1% crystal violet (Sigma, Germany, #109218) for 20 min. Cells were photographed under Leica AM6000 microscope (Leica, Wetzlar, Germany) and the number of immigrating cells from five random fields of each sample was counted [11].

### ELISA

ELISA kits were purchased from Elabscience Biotechnology Co., LTD., Wuhan, China. The inflammatory cytokines (IL-1β, IL-6, and TNF-α) from the cell culture supernatant were measured. The supernatant of cells was collected and 100 µl of the supernatant was used to measure concentrations of interleukin (IL)-1β, interleukin (IL)-6 and tumor necrosis factor (TNF)-α. Briefly, the supernatant was added to the capture-antibody-coated plate for 1 h incubation. After a washing step to remove unbound material, biotin-labeled detection antibody was added, this was followed by the addition of streptavidin–HRP chemiluminescent detection reagent. After 30 min incubation, the plate was washed 3 times with washing buffer, and the optical density of samples and standards was measured at 450 nm using a microplate reader (Infinite 200 PRO; Tecan). The samples and standards were measured in triplicates and the concentration of each cytokine was measured based on the linear regression curve of the standards.

### Tube formation assay

Tube formation assay kit (Cell Biolabs, USA) was used for in vitro angiogenesis assay. 50 μl extracellular matrix (ECM) solution was added to a prechilled 96-well culture plate and incubated at 37°C for 20 min. Cells (1 × 10^4^) in medium with 10% FBS were added to each well and incubated for 18 h. Cell morphology was observed with a phase-contrast microscope and Image J Angiogenesis Analyzer [National Institutes of Health (NIH), Bethesda, MD, USA] was used for quantification of the tube length in each sample. Five random fields of each sample were used for quantitative analysis [11].

### Statistical analysis

The significance of the difference between two groups was evaluated by Student’s t-test. Comparisons among multiple groups were analyzed using one-way analysis of variance (ANOVA) with Tukey’s post hoc test for pairwise comparison. P < 0.05 was considered to be statistical significant. Statistical analyses were performed using the GraphPad Prism 5 software (San Diego, CA).

## Results

In this study, we investigated the functional roles of circ_0001897 in high glucose (HG)-induced inflammation and angiogenesis in human retinal microvascular endothelial cells (HRECs). HG treatment caused the upregulation of circ_0001897 in HRECs, and enhanced cell proliferation, inflammatory responses as well as *in vitro* angiogenesis. Circ_0001897 knockdown significantly attenuated cell proliferation, inflammatory responses, and angiogenesis induced by HG treatment. We further showed that circ_0001897 sponges mir-29c-3p, which in turn regulates the expression of the downstream target TGFB2. Collectively, our data suggest that circ_0001897/mir-29c-3p/TGFB2 axis is involved in the regulation of HG-induced inflammation and angiogenesis in DR.

### Circ_0001897 level is upregulated in DR samples and HG-treated HRECs

RT-qPCR was used to detect circ_0001897 expression level in peripheral blood samples of 22 DR patients and 20 healthy controls. The results showed that circ_0001897 was upregulated in the samples of DR patients when compared with that of the healthy controls (Figure 1(a)). To mimic the retina endothelial cell experiencing high glucose level in DR patients, we treated human retinal microvascular endothelial cells (HRECs) with medium with high glucose (30 mM, HG) for 48 h. Compared with the cells cultured with normal glucose leve (5 mM, NG), circ_0001897 was highly induced in cells treated with HG (Figure 1(b)). To validate the circular structure and the stability of circ_0001897, we quantified the level of GAPDH mRNA and circ_0001897 in the RNA samples of HRECs with RNase R treatment or mock treatment (treated with RNase-free water). GAPDH mRNA level was significantly reduced after RNase R treatment, while circ_0001897 level showed no significant change (Figure 1(c)). The data suggest that circ_0001897 is more stable than linear GAPDH mRNA. Together, these data revealed an upregulation of circ_0001897 in DR samples and HG-treated HRECs.

**Figure 1.** **Circ_0001897 is upregulated in DR patients and high glucose-induced HRECs**. (a) RT-qPCR was used to detect circ_0001897 expression level in the peripheral blood samples of 22 DR patients and 20 healthy subjects. (b) RT-qPCR was performed to detect the expression level of circ_0001897 in HRECs cultured with normal sugar (5 mM) and high sugar (30 mM) for 48 h. (c) RT-qPCR was used to detect the relative levels of circ_0001897 and GAPDH mRNA in the RNA samples of HRECs cells with or without RNase R treatment. The data represent the mean ± SEM from three experiments. Statistical analysis was performed using Mann-Whitney U Test (A) and two-tailed Student’s t test (b-c),*p < 0.05; **p < 0.01; ***p < 0.001.

### Silencing circ_0001897 expression alleviates HG-induced cellular changes

To investigate the functional role of circ_0001897 in HG-induced cell changes, we applied circ_0001897 siRNA that could significantly knockdown circ_0001897 level upon HG induction (Figure 2(a)). CCK-8 proliferation assay showed that HG treatment significantly promoted cell proliferation of HRECs, and circ_0001897 silencing suppressed cell proliferation (Figure 2(b)). Transwell migration experiment showed that HG treatment enhanced cell migration, while circ_0001897 silencing suppressed cell migration (Figure 2(c)). To examine the angiogenic potential, we performed tube formation assay upon HG treatment and circ_0001897 silencing. HG treatment enhanced the angiogenic potential of HRECs, which could be suppressed by circ_0001897 knockdown (Figure 2(d)). We also examined the inflammatory responses in the cell culture medium of HRECs cells upon HG treatment and circ_0001897 silencing. ELISA analysis showed that the levels of pro-inflammatory cytokines, such as TNF-α, IL-1β, and IL-6 were significantly induced by HG treatment, while their expression levels were decreased by si-circ_0001897 co-transfection (Figure 2(e-g)). Together, these results suggest that circ_0001897 upregulation contributes to the HG-induced cellular changes.

**Figure 2.** **Silencing circ_0001897 expression alleviates HG-induced inflammation and angiogenesis**. (a) RT-qPCR was used to detect the expression level of circ_0001897 in different groups of HRECs cells (NG, HG+si-NC, HG+si- circ_0001897). (b) CCK-8 proliferation assay in HRECs cells with different treatment (NG, HG+si-NC, HG+si-circ_0001897) for 48 h. (c) Transwell migration assay in HRECs cells with different treatment (NG, HG+si-NC, HG+si-circ_0001897). (d) Tube formation assay in HRECs cells in different groups (NG, HG+Si-NC, HG+si-circ_0001897). (e-g) The concentration of TNF-α, IL-1β and IL-6 in the cell culture supernatant of different groups of HRECs cells (NG, HG+si-NC, HG+si-circ_0001897) were detected by ELISA. The data represent the mean ± SEM from three experiments. Statistical analysis was performed using one-way ANOVA (a-g), *p < 0.05; **p < 0.01; ***p < 0.001.

### Circ_0001897 negatively regulates miR-29c-3p

To search for the downstream target miRNAs, we analyzed the sequence of circ_0001897 using Starbase database. It was found that circ_0001897 had a binding site of mir-29c-3p (Figure 3(a)). To confirm their functional interaction, we performed luciferase reporter assay using wild-type reporter (WT) or mutated reporter (MUT) in the presence of mir-29c-3p mimic or miR-NC. The results showed that mir-29c-3p mimic could inhibit the luciferase activity in the WT reporter, while no effect was observed in the MUT reporter (Figure 3a). Furthermore, RNA pull-down experiment showed that biotin-labeled mir-29c-3p probe enriched more circ_0001897 when compared with miR-NC control probe (Figure 3b). We also showed that circ_0001897 knockdown caused a significant upregulation of mir-29c-3p (Figure 3c). In addition, mir-29c-3p level was significantly lower in DR patients compared with healthy subjects (Figure 3d). Moreover, HG treatment could downregulate mir-29c-3p in HRECs (Figure 3e). Together, these data suggest that circ_0001897 sponges miR-29c-3p and inhibits miR-29c-3p activity.

**Figure 3.** **MiR-29c-3p served as a target of circ_0001897**. (a) By analyzing Starbase database, circ_0001897 sequence showed binding sites for mir-29c-3p and dual luciferase reporter assay was performed in HRECs cells using reporter with wild type or mutated binding sites in the presence of mir-29C-3p mimic or miR-NC. (b) RNA pull-down assay was performed in HRECs cells using biotin-labeled mir-29c-3p probe or miR-NC control probe. (c) RT-qPCR was used to detect the expression level of mir-29c-3p in HRECs cells after circ_0001897 knockdown. (d) The expression levels of mir-29c-3p in peripheral blood of 22 DR patients and 20 healthy subjects were detected by RT-qPCR. (e) RT-qPCR was used to detect the expression level of mir-29c-3p in HRECs cultured in normal glucose (5 mM) and high glucose (30 mM) induced 48 h. The data represent the mean ± SEM from three experiments. Statistical analysis was performed using Mann-Whitney U Test (D) and two-tailed Student’s t test (A, B, C, E), *p < 0.05; **p < 0.01; ***p < 0.001.

### Mir-29c-3p targets and downregulates TGFB2

Analysis of Starbase database found that the 3ʹUTR (untranslated region) of TGFB2 mRNA had binding sites for mir-29c-3p (Figure 4a). We next performed dual-luciferase reporter assay using WT and MUT reporter, and the results showed that compared with mir-NC, the co-transfection of mir-29c-3p mimic could inhibit the luciferase activity in WT reporter, but showed no effect in MUT reporter with mutated binding sequence (Figure 4a). Western blot analysis showed that mir-29c-3p mimic significantly reduced the protein level of TGFB2 in HRECs (Figure 4b), and RT-qPCR analysis showed that TGFB2 mRNA was highly expressed in DR patients compared with healthy controls (Figure 4c). Moreover, TGFB2 mRNA can be induced by HG treatment (Figure 4d). Overall, these findings suggest that TGFB2 mRNA is a target of mir-29c-3p.

**Figure 4.** **Mir-29c-3p targets TGFB2 mRNA**. (a) Analysis of starbase database revealed the presence of mir-29C-3p binding sites in TGFB2 mRNA 3ʹUTR, and dual luciferase reporter assay was performed in HRECs cells using reporter with wild type or mutated binding sites in the presence of mir-29C-3p mimic or miR-NC. (b) The expression levels of TGFB2 protein in HRECs transfected with mir-NC or mir-29c-3p mimic were detected by Western blot. (c) The expression levels of TGFB2 mRNA in peripheral blood samples of 22 DR patients and 20 healthy subjects were detected by RT-qPCR. (d) RT-qPCR was used to detect TGFB2 expression level in HRECs cultured with normal glucose (5 mM) and high glucose (30 mM) for 48 h. The data represent the mean ± SEM from three experiments. Statistical analysis was performed using Mann-Whitney U Test (C) and two-tailed Student’s t test (A, B, D), *p < 0.05; **p < 0.01; ***p < 0.001.

### Circ_0001897 regulates HG-induced cellular changes through miR-29c-3p/TGFB2 axis

To investigate whether miR-29c-3p and TGFB2 mediate the effects of circ_0001897, we transfected HRECs with circ_0001897 siRNA, circ_0001897 siRNA+ miR-29c-3p inhibitor, or circ_0001897 siRNA+TGFB2 expression vector. Western blot analysis showed that HG-induced TGFB2 upregulation could be suppressed by circ_0001897 silencing, and the co-transfection of anti-mir-29c-3p or TGFB2 expression vector partially rescued TGFB2 level (Figure 5a). CCK-8 proliferation assay showed that si-circ_0001897 attenuated cell proliferation induced by HG, and the co-transfection of anti-mir-29c-3p or TGFB2 vector partially rescued cell proliferation (Figure 5b). Similarly, Transwell migration assay and tube formation assay showed that the co-transfection of anti-mir-29c-3p or TGFB2 vector could partially rescue cell migration (Figure 5c) and tube formation ability (Figure 5d) upon circ_0001897 silencing. ELISA analysis of the pro-inflammatory cytokine also demonstrated that the effects of circ_0001897 silencing were abrogated by mir-29c-3p inhibitor or TGFB2 overexpression (Figure 5e-g).

**Figure 5.** **Circ_0001897 regulates HG-induced endothelial cell changes through miR-29c-3p/TGFB2 axis**. HRECs cells were treated with the following conditions: NG, HG+si-NC, HG+si-circ_0001897, HG+si-circ_0001897+ anti-mir-29c-3p, HG+si-circ_0001897+ TGFB2 expression vector. (a) Western blot was used to detect the protein levels of TGFB2 in different groups of HRECs cells. (b) CCK-8 proliferation assay in HRECs cells with different treatment. (c) Transwell migration assay in HRECs cells in different groups. (d) Tube formation assay in HRECs cells with above treatment. (e-g) ELISA was used to detect the concentrations of TNF-α, IL-1β and IL-6 in the supernatant of different groups of HRECs cells. The data represent the mean ± SEM from three experiments. Statistical analysis was performed using one-way ANOVA (a-g), *p < 0.05; **p < 0.01; ***p < 0.001.

## Discussion

In China, diabetes has become one of the main risk factors for cardiovascular diseases, with a high incidence of vascular complications [5,23,24]. At present, DR is has been recognized as one of the most common complications of diabetes that could eventually lead to blindness in diabetic patients [25]. Even though the incidence of DR has been increasing in China and worldwide, the underlying mechanisms of the pathogenesis of DR are poorly understood. Understanding the molecular mechanisms of the occurrence and progression of DR is of great clinical significance for the treatment and diagnosis.

In this study, we reported that circ_0001897 was upregulated in DR samples, which implies a functional role of circ_0001897 in DR. We further established a cell model of retina endothelial cell experiencing high glucose in DR patients by treating HRECs with high glucose. In HG treated HRECs, circ_0001897 was also heavily induced and the knockdown of circ_0001897 alleviated HG-induced cellular changes, including impaired migration ability, decreased tube formation ability, and diminished expression levels of inflammatory cytokines, such as TNF-α, IL-1β, and IL-6. CircRNAs regulate biological processes via diverse molecular mechanisms, such as functioning as RNA-binding protein isolators, nuclear transcriptional regulators or miRNA sponges [26]. Moreover, the circular nature of circRNAs makes it resistant to RNase digestion, which makes circRNAs more advantageous as biomarkers than linear RNAs [10]. Circ_0001897 has been shown to be highly expressed in the retinas of DR patients, which suggests that circ_0001897 may serve as a potential biomarker for DR.

Accumulating evidence has revealed that miRNAs are involved in the occurrence or the progression of DR **[**27–29**]**. A previous report showed that the expression of mir-29c-3p is altered in diabetic patients, suggesting that mir-29c-3p is involved in the development of diabetes **[**30**]**. In present study, we found that miR-29c-3p acts as a downstream target of circ_0001897, and circ_0001897 sponges miR-29c-3p and suppresses miR-29c-3p level. Importantly, miR-29c-3p mediates the effects of circ_0001897 in HG-induced inflammatory responses and angiogenesis, indicating that miR-29c-3p is a downstream mediator of circ_0001897.

TGFB2 has been widely demonstrated to regulate fibrosis and vascularization, which is implicated in the regulation of DR progression **[**31**]**. In our study, we identified TGFB2 as a target of miR-29c-3p. miR-29c-3p binds to the 3’ UTR of TGFB2 mRNA and suppresses its expression. Importantly, mir-29c-3p inhibitor or TGFB2 overexpression abrogates the effect of circ_0001897 silencing. These data suggest that circ_0001897/mir-29c-3p/TGFB2 axis regulates high glucose-induced endothelial dysfunction in DR patients.

Our study also hints several questions to be addressed. First, the mechanisms underlying the circ_0001897 dysregulation in DR patients remain to be investigated. Furthermore, the role of circ_0001897/mir-29c-3p/TGFB2 axis in DR progression should be further evaluated in animal model. Also, we observed a difference of BMI between the DR patients and healthy controls, in future work DR patients and healthy controls with similar BMI should be compared to exclude this confounding factor.

## Conclusion

In summary, we demonstrated that circ_0001897 is upregulated in DR patients as well as in HG-induced HRECs. Silencing circ_0001897 mitigates HG-induced inflammatory responses and angiogenesis in HRECs cells. We further revealed that mir-29c-3p and TGFB2 are the downstream mediators of circ_0001897. Understanding the mechanism of circ_0001897 deregulation in DR patient could provide insights into the development of novel therapeutic strategies.

## Supplementary Material

Supplemental Material
